The article "A Smart Device for a Preliminary Dental Examination Based on the Internet of Things" was retracted in 2024. Reasons: suspected computer-generated content; unreliable results or conclusions; concerns about the data; concerns about the citations.

# A Smart Device for a Preliminary Dental Examination Based on the Internet of Things

**DOI:** 10.1155/2022/7190751

**Published:** 2022-07-12

**Authors:** Mohammad Wedyan, Ryan Alturki, Foziah Gazzawe, Enas Ramadan

**Affiliations:** ^1^Department of Autonomous Systems, Faculty of Artificial Intelligence, Al-Balqa Applied University, Al-Salt 19117, Jordan; ^2^Department of Information Science, College of Computer and Information Systems, Umm Al-Qura University, Makkah, Saudi Arabia; ^3^Department of Computer Science, Prince Abdullah Bin Ghazi Faculty of Communication and Information Technology, Al-Balqa Applied University, Al-Salt 19117, Jordan

## Abstract

The COVID-19 pandemic has threatened the lives of many people, especially the elderly and those with chronic illnesses, as well as threatening the global economy. In response to the pandemic, many medical centers, including dental facilities, have significantly reduced the treatment of patients by limiting clinical practice to exclusively urgent, nondeferred care. Dentists are more vulnerable to contracting COVID-19, due to the necessity of the dentist being close to the patient. One of the precautions that dentists take to avoid transmitting infections is to wear a mask and gloves. However, the basic condition for nontransmission of infection is to leave a safe distance between the patient and the dentist. This system can be implemented by using an Arduino microcontroller, which is designed as a preliminary device by a dentist to examine a patient's teeth so that a safe distance of three meters between the dentist and the patient can be maintained. The project is based on hardware and has been programmed through Arduino. The proposed system uses a small wired camera with a length of five meters that is connected to the dentist's mobile or laptop and is installed on a robotic arm. The dentist can control the movement of the arm in all directions using a joystick at a distance of three meters. The results showed the effectiveness of this system for leaving a safe distance between the patient and the dentist. In our future work, we will control the movement of the arm via Bluetooth, and we will use a wi-fi-based camera.

## 1. Introduction

The Internet of things (IoT) has pervaded most parts of human existence in recent years, including organizations, hospitals, cities, residences, universities, industrial companies, and healthcare facilities [1]. IoT is a concept that expresses the idea of various physical devices connected to the Internet and the ability of each device to identify itself to other devices. This allows objects to be sensed and controlled remotely through the existing network infrastructure and thus creates many opportunities for the seamless integration of computer-based systems into the physical world [2, 3]. There are numerous applications that are executed in the IoT environment to carry out smart facilities and services [4].

IoT applications are enabled by technologies including wi-fi, Zigbee, Bluetooth, Internet protocol, artificial networks, artificial intelligence, smart sensors, barcodes, electronic product codes, near field communication, and radio frequency identification (RFID), among others.  Figure 1 illustrates some of these [5].

One of the most appealing application sectors for the IoT is medical and health care. Many medical applications such as remote health monitoring, senior care, chronic disease management, and fitness regimens could be enabled by the IoT to enhance access to care, reduce clinic visits, improve care quality, and, most crucially, lower the cost of care [6]. As a result, medical equipment, sensors, and diagnostic and imaging devices can all be considered smart devices or items that are integral to the IoT [7, 8].  Figure 2 depicts a number of IoT-enabled medical devices [9]. In light of the spread of COVID-19, the need to use IoT-based devices has increased in the medical field.

The coronavirus disease 19 (COVID-19) era is significant from a number of perspectives, ranging from global health to the many socioeconomic consequences [10]. Everyday behaviours have drastically changed, and people from all walks of life, especially those connected to the health sector, have been and will continue to be affected by this required transformation [11]. Unfortunately, the COVID-19 pandemic will not be stopped instantly, and everyone will have to deal with very long working and social recuperation times [12].

More than two years have elapsed since the COVID-19 pandemic began, and the SARS-CoV-2 virus and its variants have been detected in the United Kingdom, South Africa, Brazil, the United States of America, and India, among other places [13, 14]. New developing virus varieties indicate that countries are still at risk, even if they appear to have the infection under control [12]. Human-to-human transmission continues to take place via airborne droplets, direct mucosal contact, or contact with contaminated surfaces [15].

Around the world, many medical centers, especially dental facilities, have drastically decreased patient treatment by limiting clinical practice exclusively to nondeferrable urgent care [16, 17]. Dentists are more vulnerable to infection with COVID-19, due to the need for the dentist to be close to the patient to examine them. Dentists, therefore, find it difficult to keep a safe distance from their patients and have a high exposure to airborne droplets [18]. For this reason, we must take advantage of the Internet of things (IoT) to reduce the chances of transmission of COVID-19 disease between dentists and patients by maintaining social distancing as much as possible [19]. This leads us to a major research question, which is can the Arduino microcontroller device help dentists maintain a safe distance during the initial examination between the dentist and the patient?

## 2. Research Question

This research proposes a new technique for maintaining a safe distance between a dentist and patient and preventing the spread of disease by building a device that allows dentists to conduct preliminary examinations from a 3-meter distance. In light of that, one key research question is formulated: Can this device maintain a safe distance during the initial examination between the dentist and the patient?

## 3. Study Description

One effective solution to reduce the spread of COVID-19, the disease that has terrified the world and continues to threaten human lives, is for individuals to socially distance themselves as much as possible. Dental clinics are one of the most common places where the virus is spread among people, and dentists are among the people most vulnerable to infection with this virus. Many people visit dental clinics, but within some of these clinics, the service that the patient wants is not available, or the dentist is not specialized in the field of service requested by the patient. In these cases, their visit was completely unnecessary.

For example, a man visits a dental clinic and asks the dentist to adjust his teeth using porcelain veneers to improve his smile. However, he has COVID-19 at the time of his visit. When the dentist approaches the patient and examines him, the dentist finds the patient needs to go to an orthodontist (a specialized dentist in orthodontics) because this dentist is not an orthodontist and cannot provide the service the patient requires.  Figure 3 shows the patient's teeth [20]. In this case,

1. The proximity of the dentist to the patient is the reason for transmitting COVID-19 to the dentist
2. The patient's need was not met, and his visit was totally unnecessary

To avoid situations such as the one described above, in this study, we designed a preliminary examination device that allows the dentist to be 3 meters awayfrom the patientduring the examination. This examinationis a preliminaryexamination to assesswhether or not the dentistis able to meet thepatient's needs. If the preliminaryexamination shows the dentist is able to treat the patient, the dentist approaches the patient wearing latex gloves, a face shield, a head cap, and a mask, and then, the dentist treats them [21]. But if the patient's need is not within the competence of the dentist, there is no need for the dentist to approach the patient. The main goal is to achieve as much social distancing as possible between the dentist and the patient in the dental clinic on the occasions when the dentist is unable to meet the patient's need. The following section shows the components of the system.

## 4. The Components of the System

After describing the study and the main problem in the previous section, in this section, we will show all the components used in the design of our device. This system is made up of eight electronic components.  Table 1 presents these components.

The next section describes how the device is designed and its connections. It also presents the pseudocode and explains how the device works.

## 5. System Implementation

After we have presented the components of the device, we will address the device connections, the pseudocode, and how the device works.

This project involves making a robotic arm consisting of two servo motors that are controlled by a joystick using an Arduino so that the first servo moves up and down and the second servo moves right and left. A mobile is installed at the top of the robotic arm so that the front camera of the mobile is activated, and a live broadcast of what the mobile camera shows is transmitted to the dentist's laptop. The dentist controls the robotic arm using the joystick and moves it inward in different directions (up, down, left, and right). The patient opens his mouth and places it in front of the mobile without touching anything. The doctor's laptop and joystick are located three meters from the robotic arm holding the mobile phone.

To transfer the live broadcast of the patient's teeth using the mobile phone to the dentist's laptop:

1. The program “DroidCam Client” is downloaded on the dentist's laptop through https://droidcam-client.ar.uptodown.com/windows and on the mobile that is installed on the robotic arm from Google Play
2. Turn on the program on both device laptop and mobile phone
3. Click on connect button on the program that is installed on the laptop
4. The dentist starts to control the joystick, therefore moving the mobile phone that is installed on the robotic arm

Our project's design is shown in Figure 12.

To draw and simulate this project, we utilized the fritzing application, which you can get from here (https://fritzing.org/download/).  Figure 13 displays the pseudocode of our system. The next section shows the results of this device.

## 6. Results

The previous section described the project and its components and mechanisms. This section presents the results of the study.

In this research, we designed a device that could be used by a dentist to examine a patient's teeth so that a safe distance of three meters can be maintained between the doctor and the patient. To use the device, the patient opens their mouth in front of a mobile phone camera which is installed on a robotic arm. The camera can be moved in all directions by the dentist using a control device.

To do this experiment, we utilized Arduino software, which can be obtained and downloaded from https://www.arduino.cc/en/guide/windows. Arduino is programmed using the joystick's sequential readings. The robotic arm works based on the joystick reading.  Figure 14 displays the output window of the serial monitor, which shows the joystick reading and robotic arm movement.

Reminder: the robotic arm is consisting of two servos, the first servo installed on the top and the second servo on the bottom (see Figure 7).

Four levels of programming are used to program the Arduino:

) (1Level (1) (joystick_reading_of_X_axis >550): the second servo moves towards the right
) (2Level (2) (joystick_reading_of_X_axis <450): the second servo moves towards the left
) (3Level (3) (joystick_reading_of_Y_axis >600): the first servo moves down
) (4Level (4) (joystick_reading_of_Y_axis <450): the first servo moves up

What distinguishes our project is that it is unique and the first Arduino device that is based on maintaining a safe distance between the doctor and the patient in order to preserve both of their safety and to reduce the spread of COVID-19. These results proved the effectiveness of the device and that the device is working at 100%. The next section presents the conclusion of this paper.

## 7. Conclusion

A smart device for a preliminary dental examination based on the Internet of Things has been invented that allows dentists to maintain a safe distance of three meters from their patients. This project involves using an Arduino to build a robotic arm with two servo motors that are controlled by a joystick. A mobile phone is placed on the top of the robotic arm, and the phone's front camera is activated so that a live broadcast of what the camera sees is sent to the dentist's laptop. The dentist can then move the robotic arm with the joystick and move it inside the patient's mouth in various directions (up, down, left, and right). This system reduces direct contact between the dentist and the patient in situations where the dentist is unable to provide a service to the patient. Based on the results that were presented, the device has proven 100% effective and successful in maintaining a safe distance between the dentist and the patient when conducting an initial examination of the patient. Finally, we concluded that we created a simple project. Moreover, we can extend this project by using Bluetooth to control arm movement instead of a wired connection and using a wi-fi-based camera.

## Figures and Tables

**Figure 1:** IoT-based technologies [5].

**Figure 2:** IoT medical devices [9].

**Figure 3:** A patient's teeth need orthodontics [20].

**Figure 4:** Arduino UNO board.

**Figure 5:** Breadboard.

**Figure 6:** Joystick.

**Figure 7:** Robotic arm.

**Figure 8:** Male-female jumper wires.

**Figure 9:** Cable.

**Figure 10:** Servo motor.

**Figure 11:** Camera.

**Figure 12:** Project design.

**Figure 13:** A pseudocode of our system.

**Figure 14:** The output window.

**Table 1:** Device components.

NO.	Name of component	The task of the components in the device
1	Arduino UNO board, Figure 4 [22]	This piece is considered to be the basis of the project, and it is this on which any electrical project that comes to the human mind is built.
2	Breadboard, Figure 5 [22]	A breadboard is a solderless tool used to test circuit layouts and model-wide equipment. Most electronic sections in electronic circuits can be coupled by inserting their leads or terminals into the apertures and then forming connections with wires where appropriate.
3	Joystick, Figure 6 [23]	This joystick is a component that communicates directly with the user by issuing commands to move the robotic arm right, left, backward and forward. Each analog channel (axis) can have values ranging from 0 to 1023. The value of analog is roughly 512 when the joystick is in the center position. It is used to control the movement of the arm in all directions.
4	Robotic arm, Figure 7 [24]	The robotic arm consists of two servo motors. The robotic arm can be moved along the *X* and *Y* axis in both negative and positive (2-D) using a joystick.
5	Male-female jumper wires, Figure 8 [9]	Male-female jumper wires are used to connect all components with UNO.
6	Cable, Figure 9 [9]	This cable is used to link a computer with UNO.
7	Servo motor, Figure 10 [25]	This piece is the basis of the movement of the arm in all directions.
8	Camera, Figure 11 [8]	A 5-meter wired camera is installed on the head of the robotic arm and is connected to the dentist's phone or laptop.

## Data Availability

The data used to support the findings of this study are available from the corresponding author upon request.
